# Authenticated Key Agreement with Rekeying for Secured Body Sensor Networks

This article has been retracted.

**DOI:** 10.3390/s110605835

**Published:** 2011-05-31

**Authors:** Mohamed Hamdy Eldefrawy, Muhammad Khurram Khan, Khaled Alghathbar, Ahmed Saleh Tolba, Kyngn Jung Kim

**Affiliations:** 1 Center of Excellence in Information Assurance, King Saud University, P.O. Box 92144, Riyadh 11653, Saudi Arabia; E-Mails: meldefrawy@ksu.edu.sa (M.H.E.); kalghathbar@ksu.edu.sa (K.A.); ahmedtolba@ksu.edu.sa (A.S.T.); 2 Information Systems Department, College of Computer and Information Sciences, King Saud University, Riyadh, 11653, Saudi Arabia; 3 Department of Child Development & Welfare, Woosuk University, Jeonbuk, 565-701, Korea; E-Mail: kkjung00@hanmail.net (K.J.K.)

**Keywords:** body sensor network, RSA, DHECC, rekeying

## Abstract

Many medical systems are currently equipped with a large number of tiny, non-invasive sensors, located on, or close to, the patient’s body for health monitoring purposes. These groupings of sensors constitute a body sensor network (BSN). Key management is a fundamental service for medical BSN security. It provides and manages the cryptographic keys to enable essential security features such as confidentiality, integrity and authentication. Achieving key agreement in BSNs is a difficult task. Many key agreement schemes lack sensor addition, revocation, and rekeying properties, which are very important. Our proposed protocol circumvents these shortcomings by providing node rekeying properties, as well as node addition and revocation. It proposes a key distribution protocol based on public key cryptography—the RSA (Rivest, Shamir and Adleman) algorithm, and the DHECC (Diffie-Hellman Elliptic Curve Cryptography) algorithm. The proposed protocol does not trust individual sensors, and partially trusts the base station (hospital). Instead of loading full pair-wise keys into each node, after installation our protocol establishes pair-wise keys between nodes according to a specific routing algorithm. In this case, each node doesn’t have to share a key with all of its neighbors, only those involved in the routing path; this plays a key role in increasing the resiliency against node capture attacks and the network storage efficiency. Finally we evaluate our algorithm from the BSN security viewpoint and evaluate its performance in comparison with other proposals.

## 1. Introduction

The term body sensor network (BSN) [1] was coined to represent human body sensing applications in which a number of intelligent physiological sensors are integrated into a wearable wireless BSN, which can be used for computer assisted rehabilitation and/or the early detection of medical conditions. Such applications imply that outpatients can be monitored from their homes, freeing up space in hospital beds. As there is a legal requirement to keep patients’ physiological data private, any implemented network must include strong security protocols. However, its physical characteristics make incorporating security a challenging task. The constraints on sensors make the design and operation of contemporary networks exceedingly different. The existing security mechanisms for wired and wireless networks cannot be applied to BSNs, because of the constrained energy, memory and computational capability of the latter.

Key management protocols are at the core of secure communications. The goal of key management is to establish secure links between neighbor sensors in networks to exchange their data in a multi-hop fashion. Public key schemes have many advantages, such as low communication overhead, and good storage capability and scalability. These schemes can provide simpler solutions with much stronger security strength. Several researchers [2,3] have shown that public key schemes are valid on sensor nodes. The computational cost is expected to fall faster than the cost to transmit and receive. Furthermore, next generation sensor nodes are expected to combine ultra-low power circuitry allowing for a continuous energy supply.

The protocol proposed in this paper will circumvent the shortcoming of needing to provide the rekeying of nodes that occurs with previous algorithms, as well as node addition and revocation [4,5]. Therefore, with the fast growing technology, public key schemes are no longer impractical and are expected to be widely used in the near future [3]. RSA, elliptic curve and public key cryptography are all viable options on an 8-bit CPU. The relative performance advantage of ECC point multiplication over RSA modular exponentiation is inversely proportional to processor word size and directly proportional to key size [6].

Gateways have considerably high energy resources compared to sensor nodes and are equipped with high performance processors and more memory. The base station performs network management functions in a centralized fashion; constructing the Routing-Path-Table [7] for each node, depending on the installation knowledge. In location based routing, nodes are addressed by means of their locations [8]. We assume that each sensor has direct communication with the base station during key management operations, *i.e.*, the formation phase. Consequently, we will analyze the security strength of our proposal with many desirable security attributes to infer its success; our algorithm will also be compared with previous studies to evaluate its performance behavior.

The rest of this paper is organized as follows: Section 2 discusses the related work, Section 3 discusses the system architecture, Section 4 proposes our new algorithm, Section 5 evaluates the security properties, Section 6 analyzes our scheme’s performance, and finally, Section 7 concludes the paper and illustrates the future research.

## 2. Related Work

The following section discusses some of the published BSN authentication and key agreement schemes. Topics related to BSN efficiency and its shortcomings according to the desirable security attributes that will be discussed below will also be illustrated. Pre-loaded symmetric shared keys are used in large scale sensor networks for geographical region observations [9,10]. In these techniques, a certain key is loaded in each node and used to derive a shared secret key. Balfanz *et al.* [11] utilized a secure-limited channel (e.g., infrared) to exchange public-keys between parties prior to the authentication process. However, this approach requires huge resources, which would be difficult to provide in medical environments. Human confirmation of correct association is also difficult when based on public-keys and without visual cues. The resurrecting duckling protocol [12] establishes a master-slave relationship between devices whereby the first device in contact with a sensor becomes its master and can upload policies to the sensor that permits interactions with other devices. Sensors from previous patients have to be explicitly disassociated by the master before they can be reused by other patients, which may not always be practical in hospitals.

Jiang *et al.* [13] use self-certified keys (SCK) and Elliptic Curve Cryptography (ECC) to establish pair-wise keys for authentication. Each sensor agrees upon a secret with the user based on the secret information pre-loaded by a key distribution centre (KDC). Authentication is achieved if the user demonstrates knowledge of the shared secret-key with at least *t* sensors. To achieve a sensor to patient association, each patient’s BSN would require different ECC curve parameters (as each BSN is a domain), which would be impractical for the hundreds of BSN in a hospital. SNAP [14] also uses ECC to establish pair-wise keys between nodes and the gateway. It requires that each sensor be equipped with a biometric device to authenticate the patient and uses the shared secret to communicate with the base station. However, it does not establish group keys. Many studies have been conducted to address ECC-based public-key cryptography [15]. It has been found to be viable for resource constrained wireless sensor networks, providing better key distribution, management and authentication.

In a medical environment, those techniques are not sufficient, as the wireless domains of groups may overlap and only the correct sensors must be associated with each patient. Hence, the rekeying property regarding node addition and revocation is not applicable for these protocols. In addition, the pair-wise key agreement approach can’t provide resiliency against node capturing attacks and also has storage efficiency issues. From that regard our protocol has to provide the rekeying feature with key addition and key revocation options, as well as consider the storage efficiency and resiliency by the utilization of a specific routing algorithm in the key agreement process.

## 3. The System Architecture

The network topological structure is illustrated in Figure 1. The network includes gateway and sensor nodes. A gateway is less energy constrained and tamper resistant, as compared to other nodes. Sensor nodes can communicate with each other. The gateway is assumed to be secure and trusted by all nodes in the network, as soon as nodes have been loaded. Upon the knowledge of sensor nodes’ positions, the gateway begins the calculation of the routing path, considering the communication path for each node to reach the gateway hop by hop, conduct a data aggregation, and then position the network nodes with a distribution of shared session keys calculated with the cooperation of each node. The routing algorithm must be adaptive to locate alternative routing paths for each node to reach its destination, considering the trust and cost parameters of the route selections that avoid loops [16].

Involving the routing technique for the BSN provides a higher level of connectivity with a relatively small number of neighbor-shared keys. Compared with a pair-wise key distribution [17], this algorithm has to obtain an optimal routing path without considering the necessity of a mesh implantation topology, hence, by analogy, the fully mesh connected regular network is equal to the pair-wise key distribution BSN linking. According to a specified routing algorithm, each node doesn’t have to share a key with all radio-range neighbors, only those involved in the routing path.

## 4. Proposed Protocol Description

Some researchers have previously shown that with an accurate design, the widely used RSA public key cryptosystem [18] and DHECC key agreement techniques [19] can be deployed on even the most constrained of current sensor network devices. Watro *et al.* [20] proposed a mechanism for providing authentication and key exchange based on the well-known RSA cryptosystem, using *e* = 3 as the public exponent for MICA1 Motes [21]. These devices carry an Atmel ATmega 128L microcontroller with a CPU of 4 MHz of 4 KB RAM and 128 KB flash memory. The security properties of the Low Exponent variant of RSA have been studied thoroughly [22]. The proposed protocol notations are mentioned in Table 1.

The proposed key agreement protocol is provided in Table 2 which is explained as follows:

### 4.1. Key Pre-Loading Phase

The gateway is loaded with its public and private keys of the RSA cryptosystem, which means that *m* and *e* are the Gateway public keys, and *d*, such that *ed* ≡ 1mod*ϕ*(*m*) is the gateway’s private key. In addition, the gateway is loaded with the public keys of all sensor nodes *y_i_*. Each sensor node is loaded with its DHECC private key *x_i_* and the public keys of the gateway *m* and *e*.

### 4.2. Key Establishment Phase

**Step 1:** All sensors generate an ephemeral random key *r_i_*, concatenate it with *id_i_* and encrypt the result with the gateway public key to obtain (*r_i_* || *id_i_*)*^e^* mod *m*. We assume that each sensor begins the session with maximum transmission power to reach the gateway.

**Step 2:** The gateway decrypts the received vectors coming from all sensors with its private key (*r_i_* || *id_i_*)*^ed^* ≡ (*r_i_* || *id_i_*)mod *m* to obtain *r_i_* for each *S_i_*. According to the routing map, after the gateway has been calculated, it starts to send the session keys to each node, as shown in Figure 1. The nodes *S*_1_, *S*_2_, *S*_3_, and *S*_4_ are from the same cluster *P_I_*, and as such, they will obtain the same session key.

**Step 3:** The gateway responds to these nodes by sending 𝒵_*P*_*I*__ = *G*(*r*_*S*_1__ + *r*_*S*_2__ + *r*_*S*_3__ + *r*_*S*_4__) encrypted by the DH long term private key for each node. For example, node *S*_1_ will receive *y*_*S*_1__(*r*_*S*_1__ + *r*_*S*_2__ + *r*_*S*_3__ + *r*_*S*_4__), from the gateway and then *S*_1_ will calculate 𝒵_*P*_*I*__ = (*y*_*S*_1__/*x*_*S*_1__) (*r*_*S*_1__ + *r*_*S*_2__ + *r*_*S*_3__ + *r*_*S*_4__). As such, we realize that many nodes can share more than one cluster, which also means that they share more than one key. This manner of key distribution primarily depends on the routing path established by the gateway.

### 4.3. The Steady State Phase

Considering node *S*_1_ that would like to send information to the gateway through $S_{1}\overset{P_{I}}{\to }S_{2}\overset{C_{1}}{\to }S_{5}\overset{P_{II}}{\to }S_{8}\overset{P_{II}}{\to }GW$, it sends its information to node *S*_2_, encrypted with Z_*P*_*I*__. *S*_2_ then forwards it to deliver *S*_5_ encrypted with Z_*C*_1__, and *S*_5_ delivers it to *S*_8_ encrypted with Z_*P*_*II*__. Finally, *S*_8_ delivers it to the gateway encrypted with Z_*P*_*II*__. Node *S*_1_ has alternative routing paths, to be used as needed, and therefore, the established session key between nodes is used later for a symmetric encryption for secure data forwarding to the gateway.

After a random period of time, any node in the cluster could initiate the rekeying in the following two steps:

**Step 1:** *S_i_* generates another ephemeral random key *r_i_*′ and send it to the gateway in the same fashion as the second phase. In a parallel fashion, *S_i_* sends this new ephemeral key *r_i_*′ concatenated with its *id_i_* concatenated with the present ephemeral key *r_i_* to its neighbors encrypted with the shared session key between them *E*_𝒵_*Pi*__ (*r_i_*′ || *id_i_* || *r_i_*).

**Step 2:** The gateway establishes a new session key for this cluster and sends it to the cluster nodes, while the cluster nodes themselves have calculated this new key by decrypting the received vector from node *S_i_*. They can replace the old *r_i_* with the new *r_i_*′ and compare the new key that comes from the gateway with the key they have calculated to validate the integrity.

### 4.4. Key Revocation and Addition

The applicability of the additively homomorphic DHECC algorithms plays a key role in the nodes’ addition and revocation.

**The revocation:** In the case of node capturing, or when a predefined value of a node life time is reached, the gateway begins the revocation by removing the current ephemeral random key for this node from the session key shared with this node’s neighbors. The gateway then resends the new key to all neighbors encrypted with their static private key. Consequently, we consider that the gateway has the ability to detect the nodes’ capture [23].

**The addition:** Establishing a key for a new node loaded by its public and private keys, *x_i_*, *y_i_* and the gateway public key *m* = *PQ*, with the network sensor nodes is similar to Vector Exchanging and the Key Establishment Phases. We assume that the gateway is informed by the public key of the new node before node installation.

## 5. Security Analysis

The inherent security [24] relies on the difficulty of recovering this key via the factorization of large integers. It is generally accepted that RSA keys should be a minimum of 1,024 bits. Discrete logarithm cryptography (DLC) is another area of cryptography where security is provided by difficulty in solving logarithmic equations over large finite groups. Elliptical Curve Cryptography (ECC) is a subset of DLP, where the discrete logarithmic solutions occur over an equation of a plane curve. Wireless networks are more vulnerable to attacks than their wired counterparts, due to the nature of wireless transmission, resource limitations and uncontrolled environments that represent a great challenge in BSN security. BSNs have the following security requirements [25,26]:

**Known Key Security:** The protocol should still achieve its goal in the face of an adversary who has learned other session keys *Z_cj_*. Hence, each run of the protocol between the nodes and the gateway produce a unique session key that depends on the random ephemeral keys *r_i_* of nodes *S_i_*. The adversary, who learned some other session keys, can’t predict new or subsequent session keys *Z_cj_* (forward secrecy), and also can’t predict any earlier session keys (backward secrecy).

**Key Control:** Neither of the principles who share the key agreement process are able to force the key to be any chosen value, otherwise, one party could force the use of an old key, key disposable safety. One potential benefit is that each principle doesn’t have to rely on any other party to generate appropriate keys. As long as neither party is malicious, it can often be guaranteed that the session key *Z_cj_* is a sufficiently random input. A related benefit is that principals can often be sure that the session key is fresh by ensuring that their own input is fresh. Consequently, involving an ephemeral random key generated by each node *r_i_* to share the session key establishment is to grant the key freshness of the session key and provide the key control property.

**Implicit Key Authentication:** A key establishment protocol is said to provide implicit key authentication (of *S_i_* to the gateway) if the gateway is assured that no other node *S_i_*, aside from the specifically identified *S_i_*, can learn the value of a particular secret key. A key agreement protocol which provides implicit key authentication to both participating principals is called the authenticated key agreement (AK) protocol. Our algorithm implicitly authenticates the exchanged information sensor nodes and the gateway using the long term private keys of others.

**Key Confirmation:** A key agreement protocol satisfies key confirmation; if one party is assured that all other parties have possession of a particular secret key, through the rekeying process, then the new session keys established by the gateway are compared with their similar, node self generation, keys. The lack of termination means that each node has the correct key, thus, the gateway confirms that the sensor nodes possess the correct secret key. This property only covers the steady state (rekeying) phase, a very frequent process. If this isn’t the case, node addition and revocation, the sensor nodes, have to trust the gateway; this is referred to as the partial trust of the gateway.

**Explicit Key Authentication:** If both implicit key authentications and key confirmations are provided.

**Node Capture:** Each node is pre-loaded with a unique private and public key of itself, the gateway public key, and a random ephemeral session key, revealed by node capturing. In this case, they cannot provide any profit to the intruder about the network, or the rest of the nodes. Our proposal achieves a good degree of resilience against node capture, because of the key freshness.

**Scalability:** The ability to support larger networks by adding more nodes is already provided through this algorithm, as discussed previously. The key distribution mechanism supports large networks and is flexible against a substantial increase in the size of the network after installation.

**Confidentiality:** This aspect is ensured by using symmetric encryption to encrypt the exchanged traffic by the established session keys between sensors. The confidentiality is conducted using periodic key freshness to prevent long term attacks.

**Key Freshness:** The derived session key must be fresh, as opposed to the reuse of old keying material. Since sensors generate the random integer *r_i_* for each session, we guarantee the key freshness property. We can also refer to this property as the ability to resist predictable attacks.

## 6. Performance Analysis

In this section, we analyze the performance of our algorithm with respect to storage and computational costs.

### 6.1. Storage Analysis

The storage complexity is the amount of memory (RAM size) required to store security credentials. The storage complexity in turn affects the hardware cost of sensor nodes. Our proposal considers the base station as the resource-rich node. Other schemes depend on key distribution before installation, which involves a tradeoff between the numbers of keys each node must store (*storage*) and the number of secure links between the nodes in the resulting network (*connectivity*). Our proposal achieves a key agreement system after deployment, according to a routing strategy. The many-to-one traffic pattern dominates in typical sensor networks, where all sensors send data to one sink [27]. Because of the many-to-one traffic pattern, a sensor node only communicates with a small portion of its neighbors, e.g., neighbor sensors that are in the routes from itself to the sink [28,29]. This means that a sensor node does not require shared keys with all neighbors. By consulting the datasheet of the PIC Microcontroller PIC18F2550 [30], we find that it has RAM of 2 Kbytes and a ROM of 24 Kbytes, which is enough for key generation for RSA (2 Kbytes).

The implementation of the prime field algorithms used 635 bytes of RAM (data) memory and 4,072 bytes of ROM (program) memory. This accounts for approximately 31% of the RAM (data) memory and approximately 13% of the ROM (program) memory available on the microcontroller [30]. Table 3 comes from a Standard Datasheet for the microcontroller which we have used; it also shows a comparison of different microcontrollers from the same family, and highlights the most important characteristics RAM, ROM which is critical when implementing cryptography algorithms on a small microcontroller.

### 6.2. Computation Analysis

Considering the computational complexity, many studies have been conducted to address PKC for sensor networks. Gura *et al.* [31] established the elliptical curve cryptography signature verification needs of 1.62 s using 160-bit keys on ATmega 128 of 8 MHz CPU; the processor was used for a Crossbow motes platform [31]. These results illustrate that ECC-based algorithms are good to use. In addition, the protocol by Watro *et al.* [23] was implemented on MICA1 Motes [21]. These devices carry an Atmel ATmega 128L microcontroller running at 4 MHz with 4 KB of RAM and 128 KB of flash memory.

This implementation was conducted over six years ago. Currently, there are many sensor nodes with high resources [32] compared with MICA1. In our study, an implementation of an elliptic curve cryptosystem on a Microchip PIC18FXX [30] family microcontroller is outlined. We designed a simple prototype diagram for our study [33] (Figure 2).

Figure 2 shows the schematic diagram of a simple sensor node. Each node consists of an Amplitude Shift Key transmitter and Receiver with a carrier frequency of 433 MHz for transmitting/receiving digital measurement data like temperature, light, *etc.* The ASK sensor is connected through the Microcontroller by using the digital Port of the microcontroller. The Random Number Generator Circuit feeds the microcontroller with random sequences that can be used for cryptography algorithms and key exchange techniques.

We chose PIC18FXX [30] for many reasons [34]: it’s cheap, it’s widely used, it’s available at competitive prices, and it can be used easily in BSN. The 8-bit bus width along with the data memory and processor speed limitations present some additional challenges *versus* the implementation on a general purpose computer. All algorithms required to perform an elliptic curve Diffie-Hellman key have been implemented. To minimize the processing time, the hardware circuit was designed with a clock rate of 48 MHz, the maximum clock rate of the PIC18F2550 microcontroller. This microcontroller has an internal USB interface with minimal external parts required which led to a simplified design for our study.

As the PIC18F2550 microcontroller and most 8 bit microcontrollers used in BSN do not contain a random number generator, it is necessary to either obtain random numbers from another source or incorporate a hardware random number generator into the design. For cryptographic uses, it is very important that random numbers be truly random and cannot be guessed or predicted in any way. For this problem, we designed a simple circuit for generating random sequences based on the avalanche effect. The circuit shown in Figure 2 was tested to provide the random noise input to the microcontroller. The base to the emitter junction of Q1 is used as the avalanche diode in this implementation.

Figure 3 shows the circuit diagram that is used for generating random sequences using the semi-conductor characteristics of transistors. With that regard we tried to wire up a circuit diagram as shown at that figure.

The involved capacitors in those circuits are called bypass capacitors [35], to which bypass high frequency signals from the power supply 12 VDC, so that we can get a clean Direct Current voltage, because high frequency signals may affect that random circuit generator.

**Results:** The efficiency of each of the algorithms in the prime field was measured by counting the cycles used on a simulator and then verifying the results by running it in real hardware. The elliptic curve point addition, doubling, and multiplication results were calculated using the actual times from the prime field algorithms and the number required.

Assuming that the communications time is negligible, the PIC18F2550 microcontroller can perform a Diffie-Hellman key exchange in approximately 5.4 seconds (two elliptic curve point multiplications).

Table 4 shows our simulation results when we tried to implement a Diffie-Hellman Key Exchange, we have simulated each arithmetic operation like addition, subtraction to evaluate the performance on the chosen microcontroller PIC18FXX while implementing the key exchange. We computed the cycles that are consumed by the clock of the microcontroller and the time it takes to perform the arithmetic operations that are involved in the elliptic curve algorithm. After that we present a few techniques that can enhance the performance and increase the efficiency while implementing the elliptic on small microcontrollers that are usually used in body sensor networks.

**Assembly Coding Improvements:** Most of the computationally intensive sections of this implementation have been coded in assembly language, which reduces the number of inefficiencies caused by a C compiler. Additional speed and memory efficiency may be gained by hand coding the entire implementation. This is a trade off with available time and readability *versus* possible negligible performance gains.

**Speeds *versus* Memory Tradeoff:** Our implementation can be made faster by unrolling all of the loops in the software to eliminate the counts and compare those used for the looping operation. Conversely, it could also be made smaller (more memory efficient) by using recursion and additional looping. The tradeoff between speed *versus* memory should be considered in future implementations. The PIC18F2550 microcontroller is easily capable of performing an elliptical curve Diffie-Hellman key exchange. With a working time of 5.4 seconds per exchange, this type of cryptography is not suited to high speed data transfers for this particular device. For high-speed transfers, the exchanged secret may be used as the key in a symmetric cipher, such as Rijndael (as used in the Advanced Encryption Standard [37]).

**RSA Implementation:** For implementing the RSA Public-Key Encryption algorithm, we used the same configuration as in the Elliptical Curve Diffie-Hellman key: an 8 bit PIC18F2550 microcontroller, with a clock speed of 48 MHz. We measured the speed of a single block of data 512 bits key:

**Encryption:** 2 s.

**Decryption:** 120 s.

We also tested another microcontroller, the dsPIC30F3013, which is a digital signal processor microcontroller with a Microchip^©^ with a clock speed of 30 MHz.

**Encryption:** 0.2 s.

**Decryption:** 15 s.

## 7. Conclusions

In this paper, considering the BSN security based on the public key mode, we have demonstrated a novel key management scheme with rekeying. This key agreement system establishes an ephemeral session key between sensor nodes with the participation of the gateway as a trusted third party. Group key distribution is very simple and the rekey messages are also authenticated. This facilitates the efficient renewal of group keys to cater for membership changes. The proposed protocol covers the rekeying property and considers the nodes addition and revocation from the viewpoint of secured key establishment. Rekeying, node addition and revocation features are the main shortcomings of this process as compared to previous algorithms.

We achieved the security requirements without the utilization of a secure-limited channel, like in Balfanz [11], which requires huge resources. In addition, we didn’t go to the master-slave relationship, which destroys the key control property. From another viewpoint, our protocol establishes pair-wise keys between nodes according to a specific routing algorithm, instead of loading full pair-wise keys into each node. In this way, each node doesn’t have to share a key with all of its neighbors, except those involved in the routing path, which is the key role of increasing the resiliency against node capturing and storage efficiency. We also analyzed the security strength of our proposal with many desirable security attributes to deduce its success; our algorithm has been evaluated according to its performance behavior implemented with respect to many previous studies.

Particularly, we consider some of the future areas in the study of security issues in BSN as follows. Many researchers have shown that public key operations may be practical in sensor nodes. However, private key operations are still too expensive to accomplish in a sensor node. As public key cryptography can greatly ease the design of security in BSN, improving the efficiency of private key operations on sensor nodes is highly desirable [36]. The mobility of sensor nodes has a great influence on sensor network architecture and sequentially on the routing protocols. New secure routing protocols for mobile BSN are needed to be created. Multimedia sensors might not be widely utilized for BSNs now, but will likely be in the near future. Substantial differences in authentication and encryption exist between discrete applications and continuous real time application, indicating that there will be distinctions between continuous stream security and the current protocols used in BSNs. Current studies on security in WSNs focus on individual topics such as key establishment, secure routing, secure data aggregation, and intrusion detection. QoS and security services need to be evaluated together in BSN.

## Figures and Tables

**Figure 1.** The Proposed Key Agreement Protocol in Body Sensor Network.

**Figure 2.** The Schematic Diagram with the Interfaces Consideration.

**Figure 3.** The Schematic Diagram for the Random Generator Circuit.

**Table 1.** The Proposed Protocol Notation.

**Notation**	**Description**
*P*,*Q*	Two large and distinct random primes.
*m*	*PQ* multiplication such that *ϕ*(*m*) = (*P* – 1)(*Q* – 1).
*e*	1 < *e* < *ϕ*(*m*), and 1 < *e* < *ϕ*(*m*).
*d*	The multiplicative inverse of *e* mod *ϕ*(*m*).
*G*	The generating element of DHECC.
*n*	The order of *G*.
*S_i_*	Sensor node number *i*.
*r_i_*	Random integers chosen by *S_i_*.
*t_i_*	Ephemeral public keys: *t_i_* ≡ *G* × *r_i_*.
*x_i_*	The private long-term keys of *S_i_*.
*y_i_*	*S_i_* long-term public keys: *y_i_* ≡ *G* × *x_i_*.
*id_i_*	The identification of *S_i_*.
𝒵_*P*_*i*__	The shared secret for the patent number *i*.
𝒵*_Cj_*	The shared secret for the shared cluster number *j*.

**Table 2.** The Proposed Key Agreement Protocol.

***Before Installation: Key Pre-loading Phase***	

*GW*	*m* = *PQ, e, d, y_i_*
*S_i_*	*x_i_, y_i_, e, m = PQ*

***After Installation: Vector Exchanging Phase***	

*S_i_* → *GW*	(*r_i_* || *id_i_*)*^e^* mod *m*
*GW* → *S_i_*	*x_i_*𝒵*_Cj_*

***Key Establishment Phase***	

*S_i_*	𝒵*_Cj_* = *x_i_*𝒵*_Cj_*/*x_i_*

***The Steady State (Rekeying) Phase***	

*S_i_* → *GW*	(*r_i_*′ || *id_i_*)*^e^* mod *m*
*S_i_→ S′_i_*	*E*_𝒵_*Cj*__ (*r_i_*′ || *id_i_* ||*r_i_*)
*GW* → *S_i_*	*x_i_*𝒵′*_Cj_*
*S′_i_*	$Z_{Cj}\overset{?}{=}{Z^{\prime }}_{Cj}$

**Table 3.** The PIC Microcontroller PIC18F2550 Datasheet.

Device	Program Memory		Data Memory	
	Flash (bytes)	# Single-Word Instruction	SRAM (bytes)	EEPROM (bytes)
PIC18F2455	24 K	12,288	2,048	256
PIC18F2550	32 K	16,384	2,048	256
PIC18F4455	24 K	12,288	2,048	256
PIC18F4550	32 K	16,384	2,048	256

**Table 4.** The Algorithm Execution Time Efficiency.

**Algorithm**	**Cycles**	**Time**
Addition	206	17.2 uS
Subtraction	273	22.75 uS
Multiplication	15,803	1,317 uS
Modulus *p* reduction	12,790	1,066 uS
Inverse	31,280	2,607 uS
Elliptic Curve Point Addition (1 Inv, 6 Sub, 2 Mul)	64,524	5.4 mS
Elliptic Curve Point Doubling (1 Inv, 5 Sub, 4 Mul)	95,857	8.0 mS
Elliptic Curve Point Multiplication (256 EC Dbl, 128 EC Add)	32,798,464	2.73 S
